# Correlation Analysis of Chaige Qinlian Decoction and Acupuncture Combined Intervention on Prognosis of Children with Pneumonia

**DOI:** 10.1155/2021/8229251

**Published:** 2021-12-15

**Authors:** Qi Sun, Hanshu Yu, Yun Shang, Yan Cao

**Affiliations:** ^1^Chifeng University, Affiliated Hospital of Chifeng University, Chifeng 024000, Neimenggu Province, China; ^2^Department of Pediatrics, Heze Municipal Hospital, Heze 274031, Shandong Province, China; ^3^Department of Equipment, Taian Maternal and Child Health Hospital, Taian 271000, Shandong Province, China; ^4^Department of Chinese Medicine, The Fourth People's Hospital of Jinan, The Third Affiliated Hospital of Shandong First Medical University, Jinan 250031, Shandong Province, China

## Abstract

**Background:**

Traditional Chinese medicine (TCM) treatment is of great importance to improve the clinical symptoms of children with pneumonia, and this study was conducted in this context.

**Methods:**

The clinical data of 82 child patients with pneumonia admitted to our hospital from February 2019 to February 2020 were retrospectively analyzed, and the patients were divided into the conventional group and the combined group according to the parity of their admission numbers, with 41 cases each. Conventional Western medicine therapy was given to children in the conventional group, and on this basis, acupuncture combined with Chaige Qinlian decoction was performed on children in the combined group, so as to evaluate the clinical application value of combined treatment and analyze its relationship with prognosis by recording the recovery time of each symptom, serum indicators, and immune indicators.

**Results:**

Children in the combined group had significantly shorter recovery time of each symptom and lower mean CPIS scores after treatment than the conventional group (*P* < 0.001); the TCM symptom scores at T1 (1 d after treatment), T2 (3 d after treatment), T3 (7 d after treatment), and T4 (10 d after treatment) of children in the combined group were significantly higher than those in the conventional group (*P* < 0.05); various immune indicators of the combined group before and after treatment were significantly different (*P* < 0.001), and after treatment, the combined group obtained significantly higher IgG levels and lower IgA, complement C3, and complement C4 levels than the conventional group (*P* < 0.001); and there was a positive correlation between the CPIS scores and serum IL-8, IL-6, and CRP levels at the first day (*r* = 0.706, 0.712, 0.734, *P* < 0.001).

**Conclusion:**

Acupuncture combined with Chaige Qinlian decoction can effectively shorten the course of disease, reduce the levels of serum inflammatory factors, and improve the immune function of body for child patients with pneumonia. Serum IL-8, IL-6, and CRP levels in child patients can reflect the clinical prognosis, with higher levels indicating worse prognosis.

## 1. Introduction

Pediatric pneumonia is a respiratory disease caused by pathogens such as bacteria or viruses, with cough, fever, and panting as the main manifestations [1, 2], and the regular moist rales can be heard via pulmonary auscultation. The Western medicine therapy is mainly antiviral and antibacterial, and long-term application will produce drug-resistant strains, which can adversely affect the prognosis and treatment of children [3]. In recent years, with the deep research and development of traditional Chinese medicine (TCM) in pediatric pneumonia, rich experience in improving the efficacy and clinical symptoms of children have been accumulated. TCM suggests [4] that pneumonia lies in the categories such as “lung wind” and “pneumonia with dyspneic cough” and that phlegmatic hygrosis character of children is the cause of the disease. Acupuncture has the efficacy of dredging meridian, supporting healthy energy to eliminate pathogenic factors and recuperating qi and blood, which can improve the body immunity of children, reduce allergic reactions, and improve the clinical symptoms by relieving asthma, dispelling phlegm, and anti-inflammation, with the efficacy proved in treating pediatric bronchial pneumonia [5]. Chaige Qinlian decoction, which is derived from the volume IV of Zhengyin Maizhi, has been proved to have the efficacy of clearing away heat and dampness as well as clearing purging fire for removing toxin and presents good efficacy in bronchopneumonia with syndrome of damp-heat obstructing lung [6], but few reports in pediatric pneumonia have been published. Based on this, the efficacy of acupuncture combined with Chaige Qinlian decoction in treating pediatric pneumonia and correlation analysis on prognosis was further demonstrated in this study, which was summarized and reported as follows.

## 2. Clinical Information

### 2.1. Baseline Information

The clinical data of 82 children with pneumonia admitted to the department of pediatrics of our hospital from February 2019 to February 2020 were retrospectively analyzed, and the patients were divided into the conventional group and combined group according to the parity of their admission numbers, with 41 cases each.

### 2.2. Diagnosis Criteria

#### 2.2.1. Diagnosis Criteria of Western Medicine

The diagnosis criteria for pediatric pneumonia in Practical Pediatric Respiratory Medicine [7] were met; the patients had fever, cough, and panting, and X-rays of the lungs showed patchy shadows or increased texture in both lungs; and in severe cases, cyanosis and wheezing were often aggravated at night or in the morning.

#### 2.2.2. Diagnosis Criteria of TCM

Relevant diagnosis criteria in the Guidelines for Diagnosis and Treatment of Common Diseases of Pediatrics in Traditional Chinese Medicine [8] with symptoms including cough, sticky and yellowish sputum, fever, panting, and red tongue accompanied by nausea, vomiting, lack of warmth in the limbs, and pale complexion.

### 2.3. Inclusion Criteria

The inclusion criteria were as follows: the patients were 1–13 years old; the patients had the disease for the first time and did not accept other treatments; the patients had good compliance and could cooperate with the treatment; the study met the approval standards of hospital ethics committee, and family members of child patients understood the purpose and process of the experimental study and signed the informed consent; and the patients did not have the history of familial atopic diseases.

### 2.4. Exclusion Criteria for the Patients

The exclusion criteria were as follows: those with mycoplasmal pneumonia, pulmonary tuberculosis, lung tumors, and other lung lesions; those allergic to the drug used in the study; those with hematologic or infectious diseases; those with deterioration of disease and required urgent treatment; and those had received the treatment of antibiotic and glucocorticoid before enrollment.

## 3. Methods

After enrollment, fever clearance, cough suppression, asthma relieving, oxygen inhalation through the nasal tube, antiinfectious treatment and in vivo electrolyte maintaining were performed to all children, and regular disinfection was conducted to the wards every day to avoid cross-infection [9].

### 3.1. Conventional Drug Therapy

Conventional symptomatic treatment with Western medicine was performed on children in the conventional group, i.e., for patients with bacterial infection, cefuroxime sodium (NMPA approval no. H20063771; manufactured: CSPC Zhongnuo Pharmaceutical Co., Ltd.; specification: 0.5 g) was intravenously infused with 50 mg/kg each time per day; for patients with virus infection, ribavirin injection (NMPA approval no. H19993911; manufactured: Guangzhou Baiyunshan Tianxin Pharmaceutical Co., Ltd.; specification: 1 ml, 0.1 g ^*∗*^ 10 bottles/box) was administered via intravenous injection with 10 mg/kg each time per day for continuous 10 days.

### 3.2. Acupuncture Combined with Chaige Qinlian Decoction

On this basis, acupuncture combined with Chaige Qinlian decoction was given to children in the combined group with the specific steps as follows. The acupoints selected were Zusanli, Hegu, and Chize on both sides and Quchi, Kongzui and Lieque; the child patients were in the spine position for routine disinfection, then 0.25 mm ^*∗*^ 25 mm filiform needles were inserted according to their body size, the uniform reinforcing-reducing method was adopted based on their tolerance, and the needles were retained for 30 min after the arrival of qi. The acupuncture was performed once per day for continuous 10 days.

10 g of Mongolian milkvetch root, 10 g of kudzu vine root, 10 g of Chinese thorowax root, 2 g of Chinese goldthread rhizome, and 6 g of liquorice root were soaked in cool water for 20 min and decocted with water for 20 min twice into Chaige Qinlian decoction; patients less than 1 year old took half dose a day, and patients more than 1 year old took one dose a day. One dose of the decoction was 80 ml and taken orally in three split times for continuous 10 days. The aforesaid two treatments were performed at the same time.

### 3.3. Clinical Observation Indexes

After treatment, the recovery time of each symptom, including the time of cough clearance, fever clearance, tonsil hyperemia clearance, laboured breathing remission, lung rale clearance, and lesion disappearance on X-ray chest film, of patients in both groups was recorded.

TCM symptom scores: the symptoms of cough, panting, fever, excessive yellowish phlegm, and lung moist rales were scored before treatment (T0), 1 d after treatment (T1), 3 d after treatment (T2), 7 d after treatment (T3), and 10 d after treatment (T4) with the 5-point Likert scale [10], the maximum score of each symptom was 7 points, and the total score of the scale was 35 points, with higher scores indicating more serious symptoms.

Before and after treatment, 5 ml of fasting peripheral vein blood was drawn from child patients, the upper serum was taken after centrifugation, placed in the refrigerator under −20°C for standby application, and tested within 24 hours. Immunoglobulins IgG and IgA and complements C3 and C4 levels were measured by the immunoturbidimetry with the kits purchased from Shanghai Huzhen Industry Co., Ltd.; serum IL-8 and IL-6 levels were measured by the ELISA method, serum C-reactive protein (CRP) levels were measured by immunoturbidimetry with the kits purchased from Nanjing Boyan Biotechnology Co., Ltd., and the serum erythrocyte sedimentation rate (ESR) was measured with the full-automatic blood sedimentation kinetic analyzer (model: Caretium XC-A30; manufactured: Wuhan Alilu Medical Equipment Co., Ltd.).

CPIS scores: clinical pulmonary infection score (CPIS) [11] was obtained two days after admission and the first day after the end of treatment, respectively, with the items including the white blood cell count, tracheal secretions, body temperature, oxygenation, X-ray chest film, and progress of infiltration in lung, and the maximum score was 12 points, with higher scores indicating more serious condition.

### 3.4. Statistical Processing

In this study, the experimental data were statistically analyzed and processed by software SPSS 21.0, the picture drawing software was GraphPad Prism 7 (GraphPad Software, San Diego, USA), enumeration data were examined with the *X*^2^ test and expressed as (*n*(%)), measurement data were examined with the *t*-test and expressed as ($\bar{x}$ ± *s*), and differences were considered statistically significant at *P* < 0.05.

## 4. Results

### 4.1. Comparison of Symptom Recovery Time of Child Patients between the Two Groups

Children in the combined group had significantly shorter recovery time of each symptom than the conventional group (*P* < 0.001) (Table 1).

### 4.2. Comparison of TCM Symptom Scores of Children at Different Moments between the Two Groups

At T1, T2, T3, and T4, the TCM symptom scores of children in the combined group were significantly lower than those in the conventional group (*P* < 0.05) (Table 2).

### 4.3. Comparison of Immune Indicators of Children before and after Treatment between the Two Groups

Before and after treatment, various immune indicators of the combined group were significantly different (*P* < 0.001); after treatment, the combined group obtained significantly higher IgG level values and lower IgA, complement C3, and complement C4 level values than the conventional group (*P* < 0.001) (Figure 1).

### 4.4. Comparison of CPIS Scores of Children after Treatment between the Two Groups

After treatment, the children in the combined group obtained significantly lower mean CPIS scores than the conventional group (*P* < 0.001) (Figure 2).

### 4.5. Comparison of Changes in Serum Indicators of Children after Treatment between the Two Groups

After treatment, various serum indicator levels of children in the combined group were significantly lower than those in the conventional group (*P* < 0.001) (Table 3).

### 4.6. Correlation Analysis between Inflammatory Factor Levels and CPIS Scores of Pediatric Patients with Pneumonia

The correlation coefficient test proved that there was a positive correlation between CPIS scores and serum IL-8, IL-6, and CRP levels in child patients at the first day of disease course (*r* = 0.706, 0.712, 0.734, *P* < 0.001) (Table 4).

## 5. Discussion

Pediatric pneumonia, which often occurs in infants and young children, is caused by the physiological and anatomical characteristics of the respiratory system, namely, narrow trachea and bronchial lumen, small number of pulmonary alveoli, easy blockage by mucus, and other features of children [12, 13], combined with the fact that the autoimmune defense system of children is not yet developed and is prone to infection and other symptoms, the disease condition will progress rapidly and critically. Conventional Western medicine has great side effects, of which antibiotics are commonly applied to treat pneumonia, but with the yearly expansion of its application range, the pathogen resistance has increased, leading to more and more unsatisfactory therapeutic effects [14]. In recent years, many scholars have applied Chinese herbal compound in the clinical treatment of lung diseases, with significant efficacy and considerable clinical application prospects. TCM believes that the etiology of pediatric pneumonia mainly includes the internal and external causes, of which the internal causes include insufficient physique and qi, immature lung development, and weakness of righteousness and poor resistance caused by postnatal loss of nourishment in children, and the internal causes include exogenous six evils and pathogenic factors, cold-warm unbalance, exogenous pathogenic wind invading the lung, pulmonary qi blockage, and phlegm stagnation. Therefore, TCM treatment mainly focuses on releasing pulmonary qi and relieving superficies as well as purging heat and relieving asthma [15–17]. Chaige Qinlian decoction has the effects such as relieving fever and promoting fluid production to quench thirst and the pharmacological actions including antibiosis, bringing down fever, promoting bile secretion, and enhancing liver detoxification, which can effectively remove inflammatory factors in the body, thereby, improving the lung function of patients [18]. Acupuncture has the efficacy of regulating spirit, qi, and depression of five viscera, so that the qi and blood of five viscera are reconciled, thus achieving the internal concentration of mental state and peace of qi and blood [19, 20].

In this study, after implementation of acupuncture combined with Chaige Qinlian decoction in child patients with pneumonia, their recovery time of each symptom after treatment was significantly lower than that of the children who received conventional treatment, which may be the result of Chaige Qinlian decoction, in which kudzu vine root had the effects of bringing down fever and relieving muscle and promoting fluid production to sooth cough, Chinese thorowax root could alleviate depression and disperse stagnated hepatoqi and reconcile superficies and interior, and Chinese goldthread rhizome and liquorice root presented the significant sterilization and anti-inflammation effect, which could remarkably improve the clinical symptoms of child patients and actively promote the prognosis quality, with an efficacy that had been proved in treating pediatric bronchial pneumonia [21]. In current research [22], the inflammatory response stimulated by pathogens such as viruses and bacteria is considered to be the pathogenesis of pneumonia in children, leading to high expression of serum levels of proinflammatory factors such as IL-6, IL-8, and CRP in children. Modern molecular immunology believes that [23] the inflammatory response will stimulate the liver to synthesize CRP in large amounts through factors such as IL-6, so its level will be significantly higher in children with pneumonia. In this study, it was found that by implementing acupuncture combined with Chaige Qinlian decoction treatment to the children, the levels of serum inflammatory factors could be reduced, and the course of pneumonia in the children could be effectively shortened.

CPIS is currently an important assessment for the severity of pulmonary infections in patients, with higher scores indicating more severe pulmonary infections in patients. The results of relevant coefficient tests found that the levels of various serum inflammatory factors in children were positively correlated with the CPIS score, which was similar to the findings of IWATA et al. [24], indicating that the levels of serum inflammatory factors in children with pneumonia could reflect the severity of disease. Whereas IL-8 had a dual immune effect in humans, with low dose, it had the effect of defense against infections, and with overexpression, it would induce inflammatory responses, and therefore, higher expression levels of such serum factor indicated worse prognosis of the disease [25]. Shortcomings of this study: due to the limited study conditions, the number of included cases was small, case source lacked diversity, no analysis from a dosimetry perspective was conducted, and no research on toxic and side effects in child patients was carried out, so further exploration is required in the future.

In conclusion, the combination treatment of acupuncture and Chaige Qinlian decoction is a reliable plan to ameliorate various symptoms in child patients with pneumonia and shorten the course of disease, and such strategy greatly lowers their serum inflammatory factor levels. The serum IL-6, IL-8, and CRP expression levels are related to disease prognosis, so further research will be conducive to establishing a better solution for such patients.

## Figures and Tables

**Figure 1:** Comparison of immune indicators of children before and after treatment between the two groups ($\bar{x}$ ± *s*). (a) The comparison of IgG level values before and after treatment between the two groups: the horizontal axis indicates before and after treatment and the horizontal axis indicates the IgG level values in g/L; before and after treatment, the IgG level values of children in the conventional group are (5.63 ± 1.23) and (6.23 ± 1.39), respectively; before and after treatment, the IgG level values of children in the combined group are (5.63 ± 1.23) and (9.36 ± 1.47), respectively. ^*∗*^IgG level values of children in the combined group before and after treatment are significantly different (*t* = 12.461, *P* < 0.001). ^*∗∗*^IgG level values of children in both groups after treatment are significantly different (*t* = 9.906, *P* < 0.001). (b) The comparison of IgA level values before and after treatment between the two groups: the horizontal axis indicates before and after treatment and the horizontal axis indicates the IgA level values in g/L; before and after treatment, the IgA level values of children in the conventional group are (1.78 ± 0.63) and (1.64 ± 0.42), respectively; before and after treatment, the IgA level values of children in the combined group are (1.76 ± 0.62) and (1.05 ± 0.34), respectively. ^*∗*^IgA level values of children in the combined group before and after treatment are significantly different (*t* = 6.429, *P* < 0.001). ^*∗∗*^IgA level values of children in both groups after treatment are significantly different (*t* = 6.991, *P* < 0.001). (c) The comparison of complement C3 level values before and after treatment between the two groups: the horizontal axis indicates before and after treatment and the horizontal axis indicates the complement C3 level values in g/L; before and after treatment, the complement C3 level values of children in the conventional group are (2.56 ± 0.47) and (2.38 ± 0.52), respectively; before and after treatment, the complement C3 level values of children in the combined group are (2.54 ± 0.48) and (1.67 ± 0.51), respectively. ^*∗*^The complement C3 level values of children in the combined group before and after treatment are significantly different (*t* = 7.954, *P* < 0.001). ^*∗∗*^The complement C3 level values of children in both groups after treatment are significantly different (*t* = 6.242, *P* < 0.001). (d) The comparison of complement C4 level values before and after treatment between the two groups: the horizontal axis indicates before and after treatment, and the horizontal axis indicates the complement C4 level values in g/L; before and after treatment, the complement C4 level values of children in the conventional group are (1.08 ± 0.23) and (1.02 ± 0.18), respectively; before and after treatment, the complement C4 level values of children in the combined group are (1.06 ± 0.21) and (0.58 ± 0.19), respectively. ^*∗*^The complement C4 level values of children in the combined group before and after treatment are significantly different (*t* = 10.853, *P* < 0.001). ^*∗∗*^The complement C4 level values of children in both groups after treatment are significantly different (*t* = 10.764, *P* < 0.001).

**Figure 2:** Comparison of CPIS scores of children after treatment between the two groups ($\bar{x}$ ± *s*). The horizontal axis indicates the combined group and the conventional group, and the vertical axis indicates the CPIS score (points); after treatment, the mean CPIS scores of children in the combined group and the conventional group are (4.46 ± 2.03) and (6.37 ± 2.19), respectively. ^*∗*^After treatment, the mean CPIS scores of children in both groups are significantly different (*t* = 4.096, *P* < 0.05).

**Table 1:** Comparison of symptom recovery time of child patients between the two groups ($\bar{x}$ ± *s*, *d*).

Group	*n*	Fever clearance time	Cough clearance time	Tonsil hyperemia clearance time	Laboured breathing relief time	Lung rale clearance time	Time of lesion disappearance on X-ray chest film
Conventional group	41	3.81 ± 0.76	9.67 ± 2.17	6.18 ± 1.84	3.55 ± 0.74	5.17 ± 0.69	8.25 ± 1.87
Combined group	41	2.75 ± 0.85	7.03 ± 1.97	4.27 ± 1.92	2.64 ± 0.53	4.06 ± 0.73	6.53 ± 1.75
*t*		5.953	5.768	4.599	6.402	7.076	4.300
*P*		<0.001	<0.001	<0.001	<0.001	<0.001	<0.001

**Table 2:** Comparison of TCM symptom scores of children at different moments between the two groups ($\bar{x}$ ± *s*, points).

Group	*n*	T0	T1	T2	T3	T4
Conventional group	41	25.10 ± 4.68	21.36 ± 3.87	16.25 ± 2.75	9.35 ± 1.72	5.27 ± 1.65
Combined group	41	25.14 ± 4.71	18.25 ± 3.46	12.46 ± 2.89	6.53 ± 1.56	2.85 ± 1.53
*t*		0.039	3.836	6.083	7.776	6.886
*P*		0.969	<0.001	<0.001	<0.001	<0.001

**Table 3:** Comparison of changes in serum indicators of children after treatment between the two groups ($\bar{x}$ ± *s*).

Indicators	Combined group (*n* = 41)	Conventional group (*n* = 41)	*t*	*P*
IL-8 (pg/ml)	62.17 ± 5.17	75.16 ± 6.27	10.235	<0.001
IL-6 (pg/L)	36.71 ± 6.75	62.15 ± 6.26	17.695	<0.001
CRP (mg/L)	46.71 ± 4.67	72.17 ± 4.18	26.011	<0.001
ESR (mm/h)	19.28 ± 5.16	27.38 ± 5.17	7.101	<0.001

**Table 4:** Correlation analysis between inflammatory factor levels and CPIS scores of pediatric patients with pneumonia.

Indicators	CPIS	
	Correlation coefficient	*P*
IL-8	0.706	＜0.001
IL-6	0.712	＜0.001
CRP	0.734	＜0.001

## Data Availability

The data used to support the findings of this study are available from the corresponding author upon request.
